The article "Numerical simulation and mathematical modeling of biomechanical stress distribution in poroelastic tumor tissue via magnetic field and bio-ferro-fluid" was published in 2024. Journal: Heliyon.

# Numerical simulation and mathematical modeling of biomechanical stress distribution in poroelastic tumor tissue via magnetic field and bio-ferro-fluid

**DOI:** 10.1016/j.heliyon.2024.e34651

**Published:** 2024-07-15

**Authors:** Mahdi Halabian, Borhan Beigzadeh, Majid Siavashi

**Affiliations:** a Biomechatronics and Cognitive Engineering Research Lab, School of Mechanical Engineering, Iran University of Science and Technology, Tehran, Iran; b Applied Multi-phase Fluid Dynamics Lab, School of Mechanical Engineering, Iran University of Science and Technology, Tehran, Iran

**Keywords:** Magnetic force and bio-ferro-fluid, Biomechanical stress, Apoptosis, Poroelastic tumor, Numerical simulation and mathematical modeling

## Abstract

Based on scientific evidence, it seems that bio-magnetic systems can change the process of cancer cell death by affecting the distribution of pressure and mechanical stress in the tumor tissue. Already most of the research has been done experimentally and few mathematical modeling and numerical simulations have been done to investigate the relationship between the magnetic parameters and the mechanical stress of the tumor tissue. This is despite the fact that in order to be able to make new equipment with the help of medical engineering methods, it is definitely necessary that the mathematics governing the problem and changes in the effective magnetic parameters (such as the shape of the magnetic source, magnetic flux density, magnetic source distance and ferro-fluid volume fraction) should be studied as much as possible. In this research, using numerical simulation and mathematical modeling, four common geometrical shapes (rectangular and circular) of the static magnetic field source were used to investigate the relationship between the change of the effective magnetic parameters and the mechanical stress created in the tumor tissue. The results of this research showed that when the magnetic flux density and ferro-fluid volume fraction and also the distance between the magnet and the tissue are kept constant, as well as without spending any extra energy, for a rectangular magnet, just by changing the way the source is placed on the tissue, the average biomechanical stress inside the tumor tissue causes a 25 % change. Also, for a circular magnet, just by doubling the radius of the magnet, the average biomechanical stress inside the tumor tissue causes a 73 % change.

## 1 Introduction

One of the world's great thinkers has said beautifully that health clothing is one of the most beautiful clothes for humans and there is no greater calamity for man than chronic physical illness. In this regard, cancer can be considered as one of the most difficult human diseases which literally is a great tragedy for the patient and those around him. Today, unfortunately, human life style is tied to some environmental factors and high-risk habits and behaviors; Some of them include smoking and alcohol consumption [1], unprotected exposure to ultraviolet rays and other harmful electromagnetic waves [2], as well as exposure to viral infections and physical and mental damage that cause genetic and non-genetic changes; According to scientific research, these factors, in turn, provide the basis for the onset, growth, proliferation and metastasis of cancer cells [3,4]. The high prevalence of cancer in Iran and other parts of the world [5] has led to increased scientific efforts to improve the quality of treatment processes and reduce their costs. In fact, it seems that researchers should be looking for innovative methods to treat tumors and cancerous tissues that can both reduce the biological side effects and financial costs of treatment and increase the efficiency of treatment. Perhaps one of the most important methods in this field are bio-magnetic systems based on bio-magnetic carriers and magnetic fields, which due to their special features and capabilities, have received much attention today in cancer research centers [6,7]. At present, because of the discovery of new biocompatible micro/nano magnetic particles, the development of magnetic drug targeting is promising [8,9], because these particles are small enough on the one hand which can penetrate into the holes of the cell membrane and on the other hand, they are big enough which can be controlled by an external magnetic field [10]. This unique feature of bio-magnetic particles has led to the production of highly functional magnetic carriers for magnetic drug targeting. One of these widely used carriers is bio-magnetic ferro-fluids. Bio-magnetic ferro-fluids are actually colloidal suspensions of magnetic nanoparticles whose behavioral properties are different in the presence and absence of external magnetic fields. The importance of using of bio-magnetic ferro-fluids in magnetic drug delivery have led some researchers to study the improvement of rheological properties and the optimal method of using them inside the body of living organisms [11,12] and some other researchers are studying to make the equipment and discover a newer capability of them [13,14]. But maybe the most important reasons and characteristics of the use of bio-magnetic carriers and magnetic fields, as innovative methods to treat tumors and cancerous tissues, are that magnetic fields have the ability to affect on a magnetic object without direct contact with it, as well as the use of magnetic fields in a certain range is safe for living tissue; for these reasons, controlled magnetic space will have minimal side effects on biological systems, and as a result, micro/nano-magnetic carriers and specially bio-ferro-fluid can be guided within the body with minimal invasive action [15,16]. The use of magnetic properties applied in therapy (not diagnostics) has been seriously considered in the last five decades. These applications include the use of a permanent magnet to concentrate the drug-containing magnetic particles near the surface of the body [17,18]; the other application can be the use of magnetic fields for the treatment of hyperthermia, which is naturally used to increase the temperature level to destroy the cancerous mass by creating magnetic resonance in the magnetic particles [19,20]. The existence of physical limitations, low therapeutic efficacy, high cost and several side effects in the usual tumor therapeutic methods like hyperthermia, chemotherapy and surgery have led researchers to pay more attention to the physiology of cancer cells and the role of mechanical stress in cell life so that maybe can be discovered a safer and more non-invasive methods to tumor treatment.

The article "Numerical simulation and mathematical modeling of biomechanical stress distribution in poroelastic tumor tissue via magnetic field and bio-ferro-fluid" was published in 2024. Journal: Heliyon.

According to what has been mentioned, recently the research of scientists shows that cancerous cells experience various biomechanical forces in human organs, such as interaction and tensile force, compressive stresses, shear stresses, and interstitial fluid pressure [21]. In this regard, research works show that increasing the pressure inside the cancerous tissue layers causes tumor tissue compression and reduces the rate of cancer cells proliferation and growth; by expanding this compression or, by increasing the biomechanical stress around the tumor tissue, although metastasis occurs a number of them are damaged by the process of necrosis or apoptosis due to the passage of biomechanical stress beyond their tolerable range [21,22]. Among the methods that have been considered by researchers to increase mechanical stress on tumor tissue and also to encourage cancer cells to apoptosis, is the use of bio-magnetic systems and, more precisely, the use of forces caused by the magnetic field gradient [23,24]. Also, studies have shown that combining the desired properties of magnetic fields on cancer cells, considering the effect of osmotic stress due to the presence of biological fluids around tumor tissue [22], can limit tumor growth and even lead to the death of cancer cells [25,26].

By considering various research studies in the field of magnetic fields and biomechanical stress and the death of tumor cells, there are still some limitations and scientific gaps, it seems that some of the most important of them are: Firstly, the application of magnetic force and stress has been done mainly in micrometer dimensions and the stress application process in macro metric dimensions is less [27,28]. Secondly, these applications of magnetic stress are based on the paramagnetic properties of some body cells, and in cases where living cells lack this property or have little magnetic properties, applying force and magnetic stress will be limited [29,30]. Thirdly, to magnetically stimulate the cancer cells to perform the apoptosis process by existing methods, the magnetic operator must first be in direct contact with them and then to act, while direct access to some cancer cells and tumors (such as brain tumors) is not easily possible [31,32]. Fourthly, so far, most of the research has been done experimentally and few mathematical modeling and numerical simulations have been done to investigate the relationship between the magnetic parameters and the mechanical stress of the tumor tissue [33,34]. This is despite the fact that in order to be able to make new equipment with the help of medical engineering methods, it is definitely necessary that the mathematics governing the problem and changes in the effective magnetic parameters (such as the shape of the magnetic source, magnetic flux density, magnetic source distance and ferro-fluid volume fraction) should be studied as much as possible. In fact, the inherent complexities of some phenomena make it impossible to carry out experimental tests for them at the moment, or if there are, it will be very expensive. Therefore, in these cases, it may be effective to use numerical simulation methods to investigate the behavior of those phenomena. For these reasons, the main problem of this research is to know how the stress distribution in the tumor tissue due to use of magnetic field and ferro-fluid using numerical simulation and mathematical modeling. In this regard, the innovation method of this research will specifically include.

✓ Using numerical simulation and mathematical modeling, four common geometrical shapes (rectangular and circular) of the static magnetic field source are used to investigate the relationship between the change of the effective magnetic parameters (such as the shape of the magnetic source, magnetic flux density, magnetic source distance and ferro-fluid volume fraction) and the biomechanical stress created in the poroelastic tumor tissue.

The article "Numerical simulation and mathematical modeling of biomechanical stress distribution in poroelastic tumor tissue via magnetic field and bio-ferro-fluid" was published in 2024. Journal: Heliyon.

In fact, by using the innovative method introduced in this research, the gaps and limitations of the research mentioned earlier can be eliminated. In other words, in this research, it will be possible to analyze in macro metric dimensions and without considering the inherent magnetic properties of the tissue and also without direct contact with the cancer cell, the mechanical stress of the tissue can be changed by magnetic stimulation. In addition, by the innovative method of this research, after mathematical modeling of the problem, using numerical simulation, the effect of different magnetic parameters on the values of mechanical stress distribution is also evaluated. It should be noted that in this study, COMSOL Multiphysics software is selected to do numerical simulation.

## 2 Problem statement

As mentioned in the previous section, the main problem of this research is to know how to distribute stress in tumor tissue due to the use of magnetic field and ferro-fluid. Two methods of mathematical modeling and numerical simulation have been used as tools to achieve this knowledge. The reason for choosing these two methods is that, Firstly, the use of mathematical language, while providing researchers with the possibility of quantitatively examining current behaviors and also predicting future behaviors of a phenomenon, it also gives them the possibility to optimize or change or control the behaviors of that phenomenon by making or using the equipment and tools they need to achieve desired goals. For this purpose, in this research, mathematical modeling has been used to understand how stress is distributed in the tumor tissue due to use of magnetic field and ferro-fluid, under specific assumptions. Secondly, the inherent complexities and special conditions for some phenomena are such that currently, it is either simply not possible to solve mathematical models, or if there is, it will be very expensive. Therefore, in these situations, it may be effective to use numerical simulation methods to solve mathematical models and investigate the behavior of those phenomena. For this reason, numerical simulation method has been used in this research to study and evaluate the stress distribution in the tumor tissue due to the presence of magnetic field and ferro-fluid, after creating mathematical models.

Considering that all biological tissues are composed of a number of cells, the space between these cells is also filled with biological fluid, and also there is a continuous flow of fluid between blood vessels and lymph vessels with the interstitial space of cells [35,36]. Therefore, it seems that it is possible to accurately consider the living tissue environment as a porous medium with sources and sinks. In this living and porous tissue, in its natural state, two parts and physical space play the role, which are.

A) The fluid part, which includes the biological fluid in the intercellular space, as well as the blood fluid and lymph fluid in the capillary vessels.
B) The solid part, which includes the matrix part of the cell space as well as the walls of blood and lymph vessels.

The article "Numerical simulation and mathematical modeling of biomechanical stress distribution in poroelastic tumor tissue via magnetic field and bio-ferro-fluid" was published in 2024. Journal: Heliyon.

These two parts are interacting with each other. They will have effects on each other, and their final goal is to create balance and homeostasis in the living tissue. Perhaps it is possible to explain in a simple and concise way how these two parts work as follows:

Blood containing nutrients and oxygen enters through the arteries to the arterioles and then to the capillaries (source). Capillaries are the exchange of nutritious blood with tissues that this mission will be accomplished by the passage of nutrients through the capillary wall and their entry into the intercellular biological fluid and then their transfer to the wall of living cells (source). Also, these capillaries are the place of exchange of waste materials received from the tissue, which direct these materials to the venules and then to the veins (sink). On the other hand, the network of lymph vessels, while carrying out the task of transferring some substances such as hormones to the tissues, also collects and transfers part of the waste materials resulting from tissue metabolism (sink). The fluid in the network of blood vessels, lymph and the intercellular biological fluid in the porous tissue, while moving, will cause tension and pressure on the surrounding walls. Upon receiving these stresses, solid walls start to create strain on their surface that this strain change will have a mutual effect on the velocity and pressure of the flowing fluid in the fluid part.

According to what was explained above about the anatomical space and also according to the choice of method of numerical solution, as one of powerful tool to answer the problem of this research, i.e. “knowing how to distribute stress in tumor tissue due to the application and use of magnetic field and magnetic fluid”, in the following general assumptions are considered to solve the problem.

• Tumor tissue: It is the space inside the tumor that includes cancer cells, extracellular matrix, intercellular biological fluid and blood vessels. Due to some biological reasons, lymphatic vessels are not present inside the tumor [37]. This complex is considered as an elastic porous medium with flow sources. In this porous medium, the intercellular biological fluid (interstitial fluid) is assumed as the fluid part of the porous medium and cancer cells and extracellular matrix are assumed as the solid part of the porous medium and blood vessels have also been considered as the flow sources [38,39].
• Normal tissue: It is the space outside the tumor that includes non-cancerous cells, extracellular matrix, intercellular biological fluid, blood vessels and lymphatic vessels. This complex is considered as an elastic porous medium with flow sources and sinks. In this porous medium, the intercellular biological fluid (interstitial fluid) is assumed as the fluid part of the porous medium and cancer cells and extracellular matrix are assumed as the solid part of the porous medium and also blood vessels are considered as flow sources and lymphatic vessels as flow sinks [38,39].
• Capillary network: It is a network of blood vessels that surrounds the tumor and while the blood in this vascular network is a non-Newtonian fluid and is stained with bio-ferro-fluid, the vessel wall is also considered elastic [40,41].
• Although the real and biological geometry of a tumor and its vascular complex and surrounding tissue is similar to Fig. 1-A and has an irregular geometry, but to simplify the simulation process, according to concept of Fig. 1-B and 1-C, the geometry of the tumor can be considered as cylinder or sphere [39,42].

The article "Numerical simulation and mathematical modeling of biomechanical stress distribution in poroelastic tumor tissue via magnetic field and bio-ferro-fluid" was published in 2024. Journal: Heliyon.

**Fig. 1:** Physical geometry; A: 3D geometry of semi-real physic; B: cylindrical concept; C: spherical concept.
• Considering the extent and interweaving and high density of the vascular network on the tumor, to simplify the process of simulating the problem, this vascular network is considered to be integrated and actually in the form of a spherical or cylindrical layer that surrounds the tumor [43].
• The entire biological complex mentioned in the previous cases has been exposed to a static and external magnetic field [41,44].
• Using the concept of Fig. 1-B and 1-C, to perform 2D numerical simulation, the geometry shown in Fig. 2 has been used.

**Fig. 2:** A: geometry of numerical simulation. B: geometry dimensions used for simulation.
• For numerical simulation, according to Fig. 3, four different geometries are considered for the magnetic field source, which the magnetic flux density is 1.5 T for all of them. As well as volume fraction of ferro-fluid in blood is 0.5 and the distance between the center of the magnet and the center of the tissue (the tangential state of the magnet to the tissue) is assumed to be 15 mm. Horizontal and vertical rectangular magnets (H.R. and V.R. magnets, respectively) are assumed with dimensions of 10 mm × 20 mm. Also, small and large circular magnets (S.C. and B.C. magnets, respectively) are considered with radii of 5 mm and 10 mm. One of the reasons for using rectangular and circular geometrical shapes in this research is the abundance and commercial availability of these shapes of magnets [45,46].

**Fig. 3:** Different geometries used for the magnetic field source.
• In addition to the previous state, just for H.R. magnet, three others are studied for simulation, which include:
- Investigating the effect of changing the intensity of the magnetic flux density on the stress distribution in the tissue, in the magnetic flux density of 0.5, 1.5, 2, 2.5 and 3 T (which the volume fraction of ferro-fluid in blood is 0.5 and the distance between the center of the magnet and the center of the tissue is assumed to be 15 mm).
- Investigating the effect of changing the distance between the magnetic field source and the tumor tissue on the stress distribution, at distances of 15, 20, 25, 30 and 35 mm from the center of the magnet to the center of the tumor (which the volume fraction of ferro-fluid in blood is 0.5 and the magnetic flux density is 1.5 T).
- Investigating the effect of changing the volume fraction of ferro-fluid in blood on stress distribution, for values of 0.1, 0.3, 0.5, 0.7 and 0.9 (which the magnetic flux density is 1.5 T and the distance between the center of the magnet and the center of the tissue is assumed to be 15 mm).

The article "Numerical simulation and mathematical modeling of biomechanical stress distribution in poroelastic tumor tissue via magnetic field and bio-ferro-fluid" was published in 2024. Journal: Heliyon.

## 3 Governing equations

The governing equations in this research are divided into the following five categories, which are.

• Fluid [37,39,47]:

The steady state of continuity equation with sink and source of fluid in the fluidic part of the porous medium is,

(1) $$\nabla ∙\left(\varepsilon_{i}\vec{V_{i}}\right)=\left(\phi_{B}-\phi_{L}\right)\text{,}$$

Starling's law with the fluid exchange between interstitial space and the lymph vessels and blood vessels is,

(2) $$\phi_{B}=\frac{s}{\forall }L_{p}\left[\left(P_{B}-P_{i}\right)-\delta_{B}\left(\pi_{B}-\pi_{i}\right)\right]\text{,}$$

(3) $$\phi_{L}=\frac{s_{L}}{\forall }L_{p_{L}}\left[\left(P_{i}-P_{L}\right)\right]\text{,}$$

The linear momentum equation in the fluidic part of the porous medium with steady-state conditions and low velocity within porous medium and with magnetic volumetric force and neglecting the effects of fluid friction and fluid-solid phase momentum exchanges as well as the presence of a magnetic fluid (consisting of magnetic particles less than 10 nm in diameter) is,

(4) $$0=-\nabla P_{i}-\left(\frac{\mu_{i}}{k}\right)\varepsilon_{i}\left(\vec{V_{i}}-\vec{V_{t}}\right)+\varepsilon_{i}{\vec{F}}_{mag}\text{,}$$

The linear momentum equation in the blood vessels with steady-state conditions and magnetic volumetric force as well as the presence of a magnetic fluid (consisting of magnetic particles less than 10 nm in diameter) is,

(5) $$\rho_{B}\left(\vec{V_{B}}∙\nabla \right)\vec{V_{B}}=-\nabla P_{B}+\mu_{B}\nabla^{2}\vec{V_{B}}+{\vec{F}}_{mag}\text{,}$$

The steady state of continuity equation in the blood vessels is,

(6) $$\nabla ∙\left(\vec{V_{B}}\right)=0\text{,}$$

• Solid [38,48]:

The steady state of continuity equation in the solid part of the porous medium is,

(7) $$\nabla ∙\left(\varepsilon_{t}\vec{V_{t}}\right)=0\text{,}$$

The tensor of stress distribution in the solid part of the porous medium is,

(8) $${\overset{═}{\sigma }}_{total}={\overset{═}{\sigma }}_{t}+{\overset{═}{\sigma }}_{i}+{\overset{═}{\sigma }}_{B}\text{,}$$

The tensor of stress with linear elastic deformation condition is,

(9) $${\overset{═}{\sigma }}_{t}=\lambda ę\overset{═}{I}+2\mu \overset{═}{E}\text{,}$$

The tensor of stress is due to the interstitial fluid pressure is,

(10) $${\overset{═}{\sigma }}_{i}=-P_{i}\overset{═}{I}\text{,}$$

The tensor of stress is due to the presence of blood vessels on the tumor boundary is,

(11) $${\overset{═}{\sigma }}_{B}=-P_{B}\overset{═}{I}\text{,}$$

The linear momentum equation in the solid part of the porous medium with the quasi-static condition is,

(12) $$\nabla ∙\left(\varepsilon_{t}{\overset{═}{\sigma }}_{total}\right)=0\text{,}$$

The theory of infinitesimal strain in steady state and constant porosity is,

(13) $$\left\{ \begin{array}{c} ę=tr\left(\overset{═}{E}\right)=\nabla ∙{\vec{u}}_{t}\\ \overset{═}{E}=\frac{1}{2}\left(\nabla {\vec{u}}_{t}+{\left(\nabla {\vec{u}}_{t}\right)}^{T}\right) \end{array}\right.$$

(14) $$\nabla ∙\left(\vec{V_{t}}\right)=\frac{\partial ę}{\partial t}=0\text{,}$$

• Fluid-Solid [38]:

The steady state of continuity equation in the porous medium is,

(15) $$\nabla ∙\left(\varepsilon_{i}\vec{V_{i}}+\varepsilon_{t}\vec{V_{t}}\right)=\left(\phi_{B}-\phi_{L}\right)\text{,}$$

(16) $$\varepsilon_{i}+\varepsilon_{t}=1\text{,}$$

• Magnetostatic [44,47]:

Maxwell's magnetic equations in the absence of electric field and current are,

(17) $$\left\{ \begin{array}{c} \nabla \times \vec{H}=0\\ \nabla ∙\vec{B}=0 \end{array}\right.$$

Relationship between magnetic flux density and magnetic field strength and local magnetization of magnetic material as well as residual magnetic flux density is,

(18) $$\vec{B}=\mu_{0}\mu_{r}\left(\vec{M}+\vec{H}\right)+{\vec{B}}_{rem}\text{,}$$

The magnetic force is applied to the magnetic carrier is,

(19) $${\vec{F}}_{mag}=\left(\vec{M}∙\nabla \right)\vec{B}+\left(\vec{B}∙\nabla \right)\vec{M}\text{,}$$

• Numerical Boundary (according to COMSOL Multiphysics commercial software library):

Roller boundary condition used in the solid part of the porous medium is,

(20) $${\vec{u}}_{t}∙\vec{n}=0\text{,}$$

Boundary load used in the solid part of the porous medium is,

(21) $${\overset{═}{\sigma }}_{total}∙\vec{n}={\vec{f}}_{area}\text{,}$$

No flow boundary condition used in the fluid part of the porous medium is,

(22) $$-\vec{n}∙\rho_{i}\vec{V_{i}}=0\text{,}$$

The article "Numerical simulation and mathematical modeling of biomechanical stress distribution in poroelastic tumor tissue via magnetic field and bio-ferro-fluid" was published in 2024. Journal: Heliyon.

## 4 Mathematical modeling

The mathematical model introduced in this research, to calculate the total stress in the tumor tissue, is presented as follows. It is noted that Table 1 shows the nomenclature.

**Table 1:** Nomenclature.

Symbols	Unit	Explanations
$\varepsilon_{i}$	–	Volumetric fraction of the fluid part of the porous medium.
$\vec{V_{i}}$	$\frac{m}{s}$	Velocity of interstitial fluid.
$\phi_{B}$	$\frac{1}{s}$	Rate of fluid flow per unit volume, from inside of blood vessel to inside of the interstitial medium.
$\phi_{L}$	$\frac{1}{s}$	Rate of fluid flow per unit volume, from inside of the interstitial medium to inside of lymph vessel.
$\frac{s}{\forall }L_{p}$	$\frac{1}{Pa∙s}$	Filtration coefficient of the blood vessel.
$\frac{s_{L}}{\forall }L_{p_{L}}$	$\frac{1}{Pa∙s}$	Filtration coefficient of the lymph vessel.
$P_{B}$	Pa	Hydrostatic pressure of blood fluid.
$P_{i}$	Pa	Hydrostatic pressure of the interstitial fluid.
$P_{L}$	Pa	Hydrostatic pressure of lymph fluid.
$\pi_{B}$	Pa	Colloid osmosis pressure of blood fluid.
$\pi_{i}$	Pa	Colloid osmosis pressure of the interstitial fluid.
$\delta_{B}$	–	Osmotic reflection coefficient of blood components.
$\vec{V_{t}}$	$\frac{m}{s}$	Velocity of tissue.
t	s	Time.
$\vec{M}$	$\frac{A}{m}$	Local magnetization.
$\vec{B}$	T	Magnetic flux density.
$\frac{k}{\mu_{i}}$	$\frac{m^{2}}{Pa∙s}$	Hydraulic conductivity of the interstitial fluid.
k	$m^{2}$	Permeability coefficient of tissue.
$\mu_{i}$	Pa∙s	Dynamic viscosity of the interstitial fluid.
$\rho_{B}$	$\frac{kg}{m^{3}}$	Density of blood fluid.
$\rho_{i}$	$\frac{kg}{m^{3}}$	Density of interstitial fluid.
$\vec{V_{B}}$	$\frac{m}{s}$	Velocity of blood fluid.
$\mu_{B}$	Pa∙s	Dynamic viscosity of blood fluid.
$\varepsilon_{t}$	–	Volumetric fraction of the solid part of the porous medium.
ε	–	Volumetric fraction.
${\overset{═}{\sigma }}_{total}$	Pa	Total stress of the porous medium.
${\overset{═}{\sigma }}_{t}$	Pa	Stress of the solid part of the porous medium.
${\overset{═}{\sigma }}_{i}$	Pa	Stress of the fluid part of the porous medium.
${\overset{═}{\sigma }}_{B}$	Pa	Stress of tumor boundary which is due to the presence of blood vessels.
λ	Pa	Lame parameter.
μ	Pa	Lame parameter.
ę	–	Volumetric strain.
$\overset{═}{E}$	–	Strain tensor.
${\vec{u}}_{t}$	m	Tissue displacement vector.
$\vec{H}$	$\frac{A}{m}$	Magnetic field intensity.
$\mu_{0}$	$\frac{H}{m}$	Magnetic permeability of vacuum.
$\mu_{r}$	–	Magnetic relative permeability.
${\vec{B}}_{rem}$	T	Remanent magnetic flux density.
${\vec{F}}_{mag}$	$\frac{N}{m^{3}}$	Magnetic force per unit volume.
$\vec{n}$	–	Normal vector.
$J_{{\vec{u}}_{t}}$	–	Jacobian matrix.
$d_{t}$	m	Tissue diameter.
$R_{t}$	m	Tissue radius.
$d_{c}$	m	Capillary diameter.
$d_{a}$	m	Artery diameter.
$L_{t}$	m	Tissue length.
$W_{t}$	m	Tissue width.
$\rho_{t}$	$\frac{kg}{m^{3}}$	Density of solid tissue.
$P_{inlet}$	Pa	Inlet pressure.
$P_{outlet}$	Pa	Outlet pressure.
m	–	Power-law fluid model parameter.
n	–	Power-law fluid model parameter.
$L^{*}$	–	Dimensionless tissue length.
$P_{i}^{*}$	–	Dimensionless hydrostatic pressure of the interstitial fluid.
$\sigma_{total}^{*}$	–	Dimensionless total stress of the tissue.
$\sigma_{total}$	Pa	Von Mises total Stress.
L	m	Tissue length.

Considering equation (8) and using equations (10), (11), (9):

(23) $${\overset{═}{\sigma }}_{total}=\left(\lambda ę\overset{═}{I}+2\mu \overset{═}{E}\right)-\left(P_{i}\overset{═}{I}\right)-\left(P_{B}\overset{═}{I}\right)\text{,}$$

Considering equations (16), (23) as well as using equation (12):

(24) $$\nabla ∙\left(\left(\lambda ę\overset{═}{I}+2\mu \overset{═}{E}\right)-\left(P_{i}\overset{═}{I}\right)-\left(P_{B}\overset{═}{I}\right)\right)=0\text{,}$$

And using equation (13) as well as considering $\nabla {\vec{u}}_{t}=J_{{\vec{u}}_{t}}={\left(\nabla {\vec{u}}_{t}\right)}^{T}$, where $J_{{\vec{u}}_{t}}$ is the Jacobian matrix, and $\nabla ∙\left(\nabla {\vec{u}}_{t}\right)=\nabla \left(\nabla ∙{\vec{u}}_{t}\right)=\nabla^{2}\left({\vec{u}}_{t}\right)$ [38,49],:

(25) $$\left(2\mu +\lambda \right)\nabla ę-\nabla P_{i}-\nabla P_{B}=0\text{,}$$

Now by taking divergence equation (25):

(26) $$\left(2\mu +\lambda \right)\nabla^{2}ę-\nabla^{2}P_{i}-\nabla^{2}P_{B}=0\text{,}$$

Then by taking divergence equation (4) and also using equation (13)- (16), (26) and assuming

$$\varepsilon_{i}=\varepsilon_{t}=\varepsilon \text{:}$$

(27) $$\left(2\mu +\lambda \right)\nabla^{2}ę-\nabla^{2}P_{B}+\left(\frac{\mu_{i}}{k}\right)\left(\phi_{B}-\phi_{L}\right)-\varepsilon \nabla ∙{\vec{F}}_{mag}=0\text{,}$$

And also by taking divergence equation (5) and also using equation (6):

(28) $$-\nabla^{2}P_{B}+\nabla ∙{\vec{F}}_{mag}=0\text{,}$$

Finally, to calculate the total stress value from equation (8), using equations (17), (18), (25), (27), (28), It is enough to calculate the four unknowns ę and $P_{i}$ and $P_{B}$ as well as $\vec{B}$. Therefore, by solving the following equations system and assuming that other values are known, the total stress will be calculated:

(29) $$\left\{ \begin{array}{c} \left(2\mu +\lambda \right)\nabla ę-\nabla P_{i}-\nabla P_{B}=0\\ \left(2\mu +\lambda \right)\nabla^{2}ę-\nabla^{2}P_{B}+\left(\frac{\mu_{i}}{k}\right)\left(\phi_{B}-\phi_{L}\right)-\varepsilon \nabla ∙{\vec{F}}_{mag}=0\\ -\nabla^{2}P_{B}+\nabla ∙{\vec{F}}_{mag}=0\\ \left\{ \begin{array}{c} \left\{ \begin{array}{c} \nabla \times \vec{H}=0\\ \nabla ∙\vec{B}=0 \end{array}\right.\\ \vec{B}=\mu_{0}\mu_{r}\left(\vec{M}+\vec{H}\right)+{\vec{B}}_{rem}\\ {\vec{F}}_{mag}=\left(\vec{M}∙\nabla \right)\vec{B}+\left(\vec{B}∙\nabla \right)\vec{M} \end{array}\right. \end{array}\right.$$

In this research, numerical simulation is used to solve equations system (29) and for a specific geometry.

The article "Numerical simulation and mathematical modeling of biomechanical stress distribution in poroelastic tumor tissue via magnetic field and bio-ferro-fluid" was published in 2024. Journal: Heliyon.

## 5 Numerical simulation

In the numerical simulation, considering the equations presented in the previous section, blood vessels are assumed to be equivalent to the source of flow, and lymphatic vessels are equal to the sink of flow in the cellular and interstitial space. Of course, only the source of the flow is considered for the tumor tissue. It is because of biological reasons; that some lymph vessels are not present in the tumor tissue and can be omitted [37]. It should be noted that in this study, COMSOL Multiphysics commercial software is selected to do numerical simulation. To solve the equations using the finite element method, the assumed geometry is meshed with four types of elements by COMSOL Multiphysics. These four types of elements are triangle, quad, edge and vertex element. After meshing the geometry and applying the initial values, the solution of the finite element equations is calculated using Stationary solver. According to Fig. 4, in this simulation, the boundary conditions are as follows.

• The solid part of the porous medium: boundaries 1, 4 and 5 have roller boundary condition (equation (20)). Moreover, boundary 4 is assumed to have a boundary condition of the force acting on the edge (equation (21)).
• The fluid part of porous medium: boundary 1 has no flow boundary condition (equation (22)) and boundaries 4 and 5 have zero pressure boundary conditions. However, in the fluid portion of blood vessels, boundaries 2 and 3 have a pressure boundary condition, and other boundaries of blood vessels have a state of non-slip walls.

**Fig. 4:** Boundary conditions areas of numerical simulation.

The calculation algorithm in this research is shown in Fig. 5. The physical values used in this study are also shown in Table 2.

**Fig. 5:** The numerical solution algorithm used in this research.

**Table 2:** Physical values of numerical simulation.

Parameter	Value	Reference
$d_{t}$ (Tumor)	0.01 (m)	–
$R_{t}$ (Tumor)	0.005 (m)	–
$d_{c}$	0.00025 (m)	–
$d_{a}$	0.0015 (m)	–
$L_{t}$ (Healthy tissue)	0.025 (m)	–
$W_{t}$ (Healthy tissue)	0.02 (m)	–
$\varepsilon_{i}$	0.5	–
$\rho_{i}$	1020 (Kg m^−3^)	[50]
$\mu_{i}$	1.32 (Pa s)	[51]
$\rho_{t}$ (Tumor and healthy tissue)	1045 (Kg m^−3^)	[50]
λ (Tumor and healthy tissue)	91,192 (Pa)	[38]
μ (Tumor and healthy tissue)	2026.5 (Pa)	[38]
$P_{inlet}$	2080 (Pa)	[37]
$P_{outlet}$	0 (Pa)	[37]
$\rho_{B}$	1060 (Kg m^−3^)	[41]
m	0.035	[41]
n	0.6	[41]
$\mu_{r}$ (Magnet)	1	[41]
$\mu_{r}$ (Ferro-fluid)	1.3	[41]
$\frac{s}{\forall }L_{p}$ (Tumor)	42.2 × 10^−8^ ((Pa^−1^.s^−1^))	[37]
$\frac{s}{\forall }L_{p}$ (Healthy tissue)	18.9 × 10^−9^ ((Pa^−1^.s^−1^))	[37]
$\frac{s_{L}}{\forall }L_{p_{L}}$ (Healthy tissue)	1.0 × 10^−7^ ((Pa^−1^.s^−1^))	[37]
$\delta_{B}$ (Tumor)	0.82	[37]
$\delta_{B}$ (Healthy tissue)	0.91	[37]
$\frac{k}{\mu_{i}}$ (Tumor)	30 × 10^−15^ (m^2^ Pa^−1^ s^−1^)	[37]
$\frac{k}{\mu_{i}}$ (Healthy tissue)	6.41 × 10^−15^ (m^2^ Pa^−1^ s^−1^)	[37]
$\pi_{i}$ (Tumor)	1999.83 (Pa)	[37]
$\pi_{i}$ (Healthy tissue)	1333 (Pa)	[37]

The article "Numerical simulation and mathematical modeling of biomechanical stress distribution in poroelastic tumor tissue via magnetic field and bio-ferro-fluid" was published in 2024. Journal: Heliyon.

## 6 Validation

In order to verify the accuracy of the numerical solution process, it has been tried to make similar modeling using assumptions and boundary conditions in Refs. [37,38] and compare the calculation results of ę and $P_{i}$. It is noted that by using the method introduced in Ref. [38], the values of radius and pressure have become dimensionless in the form of $r^{*}=\frac{r}{R_{t}}$ and ${P_{i}}^{*}=\frac{P_{i}}{2\mu +\lambda }$, respectively. Fig. 6, Fig. 7 show the results of validation. As seen in these two figures, the results of this research are almost similar to the results of references [37,38]. The reason for the slight difference between the values is probably due to the numerical solution error or the presence of details in mentioned references that were not available. Although there is a slight difference between the values, it seems that the similarity between the results can be considered acceptable.

**Fig. 6:** Validation of volumetric strain results.

**Fig. 7:** Validation of interstitial fluid hydrostatic pressure results.

## 7 Results and discussion

As we have shown in our previous research [41], a static magnetic field can cause changes in the hemodynamic properties of a biological fluid by affecting the magnetic fluid mixed in the blood. In that study, which was merely a fluid-magnetic simulation, it was shown that the shear stress on the wall and the fluid pressure would increase or decrease by changing the geometry of the static magnetic field source. In another study [52], we showed that considering biomechanical parameters such as osmotic pressure can change the stress distribution in solid and porous tumor tissue. In that study, tumor tissue was simulated as a poroelastic model, and no volumetric force such as a magnetic force was applied to the tissue. However, it seems that according to what was discussed in the previous sections, to better understand the significance of biomechanical effects of magnetic forces and fields on the cell space, it should be considered as a volumetric force on tumor tissue. In other words, it may be better to evaluate the effect of the presence of a static magnetic force and bio-ferro-fluid on biological tissue, changes, and developments of the bio-solid part in simulations. The importance of studying the effect of static magnetic fields on biomechanical properties in the biological environment and especially the stress created in solid cellular tissue will become more apparent when it is considered that numerous studies and research on magnetic fields as a practical tool have been used to treat tumors and cancerous masses. More specifically, various studies [25,30,32] have shown that the magnetic field gradient can cause apoptosis of tumor cells by exerting pressure or stress on them and subsequently prevent them from growing and proliferating.

The article "Numerical simulation and mathematical modeling of biomechanical stress distribution in poroelastic tumor tissue via magnetic field and bio-ferro-fluid" was published in 2024. Journal: Heliyon.

To describe precisely, according to scientific findings, body cells react by changing the orientation and rearrangement of the cytoskeleton and the contractile properties of their actomyosin due to the mechanical stress applied to them. All these events are known as mechanotransduction, which represents a process during which cells receive mechanical signals and react by translating these mechanical stimulations into biochemical signals. By producing biochemical signals and interpreting them by the cell, its actions and subsequent behavior will be determined. Due to this biological capability, when living cells are exposed to the force caused by the magnetic field gradient, a mechanical stress is imposed on their plasma and walls. This mechanical stress stimulates the cellular structure and forces its internal and external components to respond biochemically or bio-electrically. Based on experimental evidence, if the mechanical stress caused by the magnetic field gradient reaches a specific and appropriate value, a living cell automatically emits a biochemical signal related to its destruction and death (apoptosis) or this mechanical stress will be so high that the whole cell is completely destroyed (necrosis). This interesting phenomenon will give this possibility to biologists and doctors which prevent the growth and proliferation of cancer cells or destroy them without using harmful chemical drugs or without performing invasive procedures and only using the mechanical stress caused by the magnetic field gradient. But because the various aspects of this interesting phenomenon are still not very clear, more research will be needed. For this reason, it has been tried in this research using numerical simulation, to help to understand more how the stress distribution in the tumor tissue due to the application and use of magnetic field and bio-ferro fluid. According to the explanation given, in the following, the results of the numerical simulation are discussed.

The article "Numerical simulation and mathematical modeling of biomechanical stress distribution in poroelastic tumor tissue via magnetic field and bio-ferro-fluid" was published in 2024. Journal: Heliyon.

Considering the geometry of Fig. 1, a combination of bio-fluid and bio-solid have been exposed to static magnetic source, as shown in Fig. 2. Of course, it should be noted that since the blood fluid in this study has ferromagnetic nanoparticles, then this fluid around the tumor can be assumed as a ferro-fluid that has been exposed to an external magnetic field. As a result, its behavior will be governed by the physical equations of ferro-hydrodynamics [47]. In the following, it will be described the results and interpretation of the numerical simulation.

According to Fig. 3, magnetic sources were placed on the tissue with a magnetic flux density of 1.5 T. Fig. 8 shows the distribution of magnetic flux density caused by these four magnetic sources in the tissue. As can be seen in this figure, since the surface of B.C. Magnet is greater than those of the other three magnets, the magnetic effect on its underlying tissue is also more significant than those caused by other magnets. Also, because S.C. Magnet has the smallest area among the other three magnets, it is seemed to have the least magnetic effect on the tissue, as shown in Fig. 9, Fig. 10. On the other hand, because circular magnets do not have sharp corners, the density distribution of the magnetic flux density within S.C. and B.C. Magnets is more uniform than the distribution of this density in the other two magnets. With a little investigation in Fig. 8, it can be seen that although the area and geometric dimensions of both H.R. and V.R. Magnets are the same, differences in the placement of the magnet on the tissue can cause a different distribution of magnetic flux density in the underlying tissue. More precisely, in the H.R. Magnet, because the contact surface of the magnet with the tissue is greater than that of the V.R. Magnet, it has a more significant magnetic effect on its underlying tissue. To investigate and compare the impact of geometrical shape on the distribution of magnetic flux density within the tumor tissue more accurately, it has been measured on the horizontal diameter of the tumor and along the circumference of its upper semicircle. Fig. 9, Fig. 10 shows this comparison. As can be seen in these figures, the highest magnetic field density created in the tumor is related to the B.C. Magnet. This difference was expected since this form of magnet has the most significant area compared to the other three magnets. The S.C. Magnet, which has the smallest the area among the other three magnets also has the lowest magnetic flux density distribution in the tumor. On the other hand, as mentioned above, the placement of the rectangular magnet on the tissue has caused the magnetic flux density distribution to be different within the tumor. More precisely, as shown in Fig. 9, Fig. 10, the H.R. Magnet has a more significant magnetic effect than the V.R. Magnet in the tumor. This difference may be due to the greater contact surface of H.R. Magnet with its underlying tissue.

The article "Numerical simulation and mathematical modeling of biomechanical stress distribution in poroelastic tumor tissue via magnetic field and bio-ferro-fluid" was published in 2024. Journal: Heliyon.

**Fig. 8:** Distribution of magnetic flux density caused by H. R. & V. R. & S. C. & B. C. Magnets in and around the tissue.

**Fig. 9:** Magnetic flux density in the tumor tissue, along its horizontal diameter by changing the geometrical shape of the magnetic field source.

**Fig. 10:** Magnetic flux density in the tumor tissue, along the circumference of its upper semicircle by changing the geometrical shape of the magnetic field source.

Considering that the blood in the peripheral capillary of the tumor is stained with ferro-fluid, Therefore, it seems that the effect of the external magnetic field on it should also be investigated. Fig. 11 shows the distribution of pressure in the vessels surrounding the tumor, both in the presence and absence of an external magnetic field. As can be seen in this figure, when an external magnetic field is applied to blood containing bio ferro-fluid, maximum pressure has arisen in the upper part of the peripheral capillary ring of the tumor, but in the absence of an external magnetic field, this maximum pressure exits the ring around the tumor and is transferred to the left branch of the capillary connected to the ring; this branch is the nearest branch to the entrance of the capillary that feeds it. According to the results of our previous research [41], the occurrence of this hemodynamic event for blood stained with ferro-fluid is expected in the vicinity of the external magnetic field. More precisely, as the magnetic fluid approaches the range of the external magnetic field, it tends to align its magnetic parts with the external source and be attracted to an external source based on Kelvin magnetic force [53] but the walls of the capillaries prevent this absorption; therefore, fluid accumulation in this part has increased and consequently increases the hemostatic pressure of the fluid. However, this does not happen in the absence of a magnetic field. In addition to what is described above, as can be seen in Fig. 8, although the position of maximum pressure is the same in all four forms, the value of this maximum is different. According to Fig. 8, Fig. 9, Fig. 10 one of the reasons for this difference is how the magnetic field density is distributed in the tissue. Changes in hemostatic pressure in the peripheral capillaries of the tumor can also cause differences in the pressure applied to the capillary wall. As a result, it is expected that this change in pressure on the vessel wall, in turn, will cause a difference in the stress distribution in the tissues around the capillaries.

The article "Numerical simulation and mathematical modeling of biomechanical stress distribution in poroelastic tumor tissue via magnetic field and bio-ferro-fluid" was published in 2024. Journal: Heliyon.

**Fig. 11:** Distribution of fluid pressure in the arteries surrounding the tumor, in the presence and absence of the magnetic field.

To study more precisely the effect of geometry change of the external magnetic field source on the pressure applied to the peripheral capillary wall of the tumor, Fig. 12 shows the pressure distribution on the upper portion of the peripheral capillary wall of it. As can be seen in this figure, the pressure distribution due to B.C. Magnet is higher than other magnets. Also, the pressure distribution due to H.R. Magnet is more than V.R. Magnet. However as mentioned, the shape and area of both H. R. and V. R. Magnets are the same, and only their placement on the tissue is different. The reason for the difference in pressure values shown in Fig. 12 can be related to the difference in the magnetic flux density values distributed around each magnet. Therefore, the higher magnetic density around the magnet and especially within its tissue and capillaries, will be caused the higher capillary blood pressure and as a result, the pressure exerted on the capillary walls. It is noted that pressure change in the absence of a magnetic field is in the form of a pressure gradient from the fluid inlet side to its outlet side but in Fig. 12, because it is displayed next to the pressure changes of other states, it can be seen almost horizontally.

**Fig. 12:** Intravascular fluid pressure on a part of tumor peripheral capillary wall, in presence and absence of magnetic field.

After investigation of the distribution of magnetic flux density and hemostatic pressure around the tumor, now the distribution of mechanical stress should be investigated within the tumor tissue. For this purpose, in four different conditions, the values of stress distribution along the horizontal diameter of the tumor and along the circumference of its upper semicircle are shown in Fig. 13, Fig. 14, Fig. 15, Fig. 16, Fig. 17, Fig. 18, Fig. 19, Fig. 20. It is noted that by using the method introduced in Ref. [38], the values of length and stress have become dimensionless in the form of $L^{*}=\frac{L}{R_{t}}$ and $\sigma_{total}^{*}=\frac{\sigma_{total}}{2\mu +\lambda }$, respectively. Fig. 13, Fig. 14 show the results of changing the shape of the magnetic field source on the mechanical stress values. Fig. 15, Fig. 16 show the results of changing the intensity of the magnetic flux density of H.R. Magnet on the mechanical stress values. Fig. 17, Fig. 18 show the results of changing in the magnetic field source distance for H.R. Magnet on the mechanical stress values. Fig. 19, Fig. 20 show the results of changing in the volume fraction of the ferro-fluid in the blood and with use of H.R. Magnet on the mechanical stress values. As seen in Fig. 13, Fig. 14, Fig. 15, Fig. 16, Fig. 17, Fig. 18, Fig. 19, Fig. 20, the amount of mechanical stress has a symmetrical pattern. More precisely, the values of stress in the areas close to the common border of the tumor and the capillaries are much higher than in the central areas of the tumor. The presence of symmetry in the circular geometry of the tumor and its peripheral capillaries, as well as the boundary conditions applied to the tumor wall, are some of the reasons that may cause this pattern. It might be said, according to equations (10), (11), (12), (13), (14), (8), (9), the central regions of the tumor are not able to move considerably compared to its outer areas and borders due to the symmetrical and dense surrounding tissue. As a result, the strain created in the central region of the tumor is much less than in the outer parts and the borders of the tumor. Because the tumor tissue is considered to be a linear elastic tissue, low strain values in the central areas of the tumor causes the relationship between stress and strain to be linear; as a result, low strain in the center of the tumor causes low stress in this area. However, by moving away from the center of the tumor and moving towards its outer wall, due to the possibility of displacement and the condition of symmetry in the porous solid boundary, the tumor tissue is can perform more displacement; therefore, the strain created in the area of the tumor wall will be much higher than its central areas. This higher strain in the areas close to the tumor wall, considering the linear relationship between stress and strain in the solid elastic tissue, causes a significant increase in mechanical stress at the tumor border.

The article "Numerical simulation and mathematical modeling of biomechanical stress distribution in poroelastic tumor tissue via magnetic field and bio-ferro-fluid" was published in 2024. Journal: Heliyon.

**Fig. 13:** Stress in the tumor tissue, along its horizontal diameter by changing the geometrical shape of the magnetic field source. Dotted lines represent the linear average of stress values.

**Fig. 14:** Stress in the tumor tissue, along the circumference of its upper semicircle by changing the geometrical shape of the magnetic field source. Dotted lines represent the linear average of stress values.

**Fig. 15:** Stress in the tumor tissue, along its horizontal diameter by changing the intensity of the magnetic flux density and for H.R. Magnet.

**Fig. 16:** Stress in the tumor tissue, along the circumference of its upper semicircle by changing the intensity of the magnetic flux density and for H.R. Magnet.

**Fig. 17:** Stress in the tumor tissue, along its horizontal diameter by changing in the magnetic field source distance and for H.R. Magnet.

**Fig. 18:** Stress in the tumor tissue, along the circumference of its upper semicircle by changing in the magnetic field source distance and for H.R. Magnet.

**Fig. 19:** Stress in the tumor tissue, along its horizontal diameter by changing in the volume fraction of the ferro-fluid in the blood and for H.R. Magnet.

**Fig. 20:** Stress in the tumor tissue, along the circumference of its upper semicircle by changing in the volume fraction of the ferro-fluid in the blood and for H.R. Magnet.

With careful in Fig. 13, Fig. 14, it can be seen that the B.C. Magnet has created the most stress in the tumor tissue. This was to be expected, given what was noted above about the higher magnetic density distribution of this magnet. In Fig. 13, Fig. 14, it can be noted that although the geometry and area of both H.R. and V.R. Magnets are the same exactly, however, the difference in their placement on the tissue has caused the stress caused by their magnetic field in the tumor tissue to make a significant difference. Of course, as mentioned in Fig. 9, Fig. 10, Fig. 12, due to the higher magnetic density distribution and the hemostatic pressure due to the presence of H.R. Magnet than V.R. Magnet, the difference in stress caused by these two magnets was also expected. In addition to what has been said, the precision in the linear average of the stress in Fig. 13, Fig. 14 is also interesting. It can be found carefully in these two figures, when the magnetic flux density and ferro-fluid volume fraction and also the distance between the magnet and the tissue are kept constant, as well as without spending any extra energy, for a rectangular magnet, just by changing the way the source is placed on the tissue, the average biomechanical stress inside the tumor tissue causes a 25 % change. Also, for a circular magnet, just by doubling the radius of the magnet, the average biomechanical stress inside the tumor tissue causes a 73 % change.

Considering Fig. 15, Fig. 16, it can be understood that, the increase or decrease of the mechanical stress in the tumor tissue is directly related to the increase or decrease of the intensity of the magnetic flux density. This relationship was also expected according to equation number (4) and equations (10), (8). It can also be seen carefully in Fig. 17, Fig. 18 that, by increasing the distance of the magnetic field source from the tissue, although the intensity of the magnetic flux density of the magnet, the geometric shape and even the way the magnet is placed in relation to the tissue have not changed in any way but the distribution of mechanical stress in the tumor tissue has decreased. Perhaps what is significant in these figures is that, as soon as the magnet moves away from the tangential position on the tissue (magnet at a distance of 15 mm), the stress distribution in the tumor is greatly reduced, which is more compared to the reduction caused by other distance changes. Perhaps the reason for this sharp decrease is that, when the magnet is in contact with the tissue, there is no air gap between the magnet and the tissue. In other words, the intermediate material between the magnet and the tumor is only healthy tissue and blood stained with biological ferro-fluid. But as soon as the magnet moves away from the tissue, the air gap is also added to the interface material between the magnet and the tumor and at longer distances, there is still air and no new material is added to these intermediate materials. And finally, according to Fig. 19, Fig. 20, it can be understood that, the increase or decrease of mechanical stress in the tumor tissue is directly related to the increase or decrease of the ferro-fluid volume fraction in the blood.

The article "Numerical simulation and mathematical modeling of biomechanical stress distribution in poroelastic tumor tissue via magnetic field and bio-ferro-fluid" was published in 2024. Journal: Heliyon.

## 8 Conclusions

In this study, a 2D numerical simulation related to the effect of static magnetic field on the mechanical stress in the porous tumor tissue was investigated. A poroelastic model was utilized to model and simulate the tumor tissue. Blood fluid and the arteries’ wall were assumed as a non-Newtonian fluid and elastic solid, respectively. Using a numerical simulation, four different geometry shapes of the source of the static magnetic field (H.R. & V.R. & S.C. & B.C. Magnets) were employed to provide an insight into the relationship between the static magnetic field and the mechanical stress created in the tumor tissue. In addition, the relation between mechanical stress with magnetic flux density as well as the distance between the magnetic source and the tissue and also changing in the volume fraction of the ferro-fluid in the blood were evaluated through this research. Considering the results of the numerical simulation showed that, when the magnetic density was kept constant, the larger geometric surface of the magnet (B.C. Magnet) caused the higher mechanical stress in the tissue. At the same magnetic density, also, a change in the placement of the magnet with respect to the tissue altered the amount of stress (H.R. and V.R. Magnets). In other word, the results of this research showed that when the magnetic flux density and ferro-fluid volume fraction and also the distance between the magnet and the tissue are kept constant, as well as without spending any extra energy, for a rectangular magnet, just by changing the way the source is placed on the tissue, the average biomechanical stress inside the tumor tissue causes a 25 % change. Also, for a circular magnet, just by doubling the radius of the magnet, the average biomechanical stress inside the tumor tissue causes a 73 % change. This study, moreover, indicated that increase of the magnetic flux density and ferro-fluid volume fraction in the blood as well as reduction of the distance of the magnetic source from the tissue increased the mechanical stress of the tumor tissue. The findings of this study disclosed that external factors such as geometrical shape of magnetic fields can considerably affect the biomechanical behavior of tumor cells, especially significant effect on the stress on the cellular scale passively. To benefit from these changes in the purpose of cancerous tumors treatment, however, more and more research is needed and the study in this important field is ongoing. In the end, in order to complete the studies carried out in this research, the following suggestions are made for future studies.

• Studying and identifying physical/chemical properties and characteristics as well as designing and manufacturing isotonic, hypotonic and hypertonic magnetic fluids according to extracellular matrix space.
• Design and construction of a magnetic device to apply external control on isotonic, hypotonic and hypertonic magnetic fluids injected into the extracellular matrix space.
• Optimizing the geometric shape of the magnetic source and the values of the magnetic flux density, the distance of the source from the tissue and the volume fraction of the ferro-fluid in the blood, in order to achieve the goal of the highest possible mechanical stress in the tumor tissue.

The article "Numerical simulation and mathematical modeling of biomechanical stress distribution in poroelastic tumor tissue via magnetic field and bio-ferro-fluid" was published in 2024. Journal: Heliyon.

## Data availability statement

No data was used for the research described in this article.

## CRediT authorship contribution statement

**Mahdi Halabian:** Writing – original draft, Visualization, Software, Methodology, Investigation, Formal analysis. **Borhan Beigzadeh:** Writing – review & editing, Supervision, Project administration, Conceptualization. **Majid Siavashi:** Writing – review & editing, Supervision, Conceptualization.

## Declaration of competing interest

The authors declare that they have no known competing financial interests or personal relationships that could have appeared to influence the work reported in this paper.
